The article "An Intelligent Optimization for Building Design Based on BP Neural Network and SPEA-II Multiobjective Algorithm" was retracted in 2023. Reasons: signs of a paper mill; suspected computer-generated content; unreliable results or conclusions; concerns about the data.

# An Intelligent Optimization for Building Design Based on BP Neural Network and SPEA-II Multiobjective Algorithm

**DOI:** 10.1155/2022/3667187

**Published:** 2022-04-22

**Authors:** Haiman Xu

**Affiliations:** Department of Art, Anhui Jianzhu University, Hefei, AnHui 230041, China

## Abstract

With the continuous development of the field of building optimization, more and more optimization methods have sprung up, among which there are many kinds of intelligent optimization algorithms. This kind of intelligent optimization algorithm usually relies on the traditional building performance simulation method to obtain the building performance index for optimization. However, intelligent optimization algorithms generally require large-scale calculations. At the same time, the time required for building performance simulation is often limited by the complexity of building models and the configuration of computers, which leads to a long time for performance optimization, which cannot give efficient and accurate feedback to designers in engineering. Building performance optimization methods based on intelligent optimization algorithms are mainly used in scientific research and are difficult to put into practical projects. Therefore, this paper builds an accurate and efficient platform for building performance prediction and optimization to help designers make decisions combined with BP neural network and the SPEA-II multiobjective optimization algorithm. Besides, the optimization results of the case are quantitatively and qualitatively analyzed and presented in visual form based on the BP neural network prediction model. Quantitative analysis includes the evolution process of solution set, convergence process, and comprehensive quality evaluation of solution set. Qualitative analysis includes Pareto frontier and optimal architectural scheme analysis. Finally, the conclusion shows that the platform prediction and optimization can give accurate and reliable optimal solution, and the optimal building scheme is reasonable and has high engineering application value.

## 1. Introduction

There are many types of public buildings, with different functions and great differences, which will be more prominent in the future. When evaluating the design scheme of public buildings, we analyzed the Chinese modern architecture and its design concept. It is very important to study how to evaluate the design scheme of public buildings and solve these problems. At present, the scheme evaluation methods adopted include the evaluation method of index system based on expert evaluation and qualitative evaluation and the method of determining the weight of evaluation indexes by the Delphi method and analytic hierarchy process (AHP), with good results. However, the main problem of AHP is that the subjective error of evaluation results caused by weighting is inevitable, and this error may be enlarged step by step with the evaluation indexes at all levels. Although there are theoretical methods to control the calculation weight error and test the evaluation result error afterwards, it is still difficult to avoid the error caused by scheme evaluation beforehand [1]. There are still some unavoidable problems when applying quantitative analysis theories and methods such as fuzzy mathematics to evaluate building schemes, mainly in determining the type of membership function, and there is no good theoretical basis to demonstrate the full rationality of the selected membership function. Therefore, the effectiveness of applying fuzzy membership function to scheme evaluation still needs further research [2]. In recent years, aiming at the problems existing in the application, a nonlinear comprehensive evaluation model that can quickly absorb the knowledge and experience of evaluation experts was designed [3, 4]. At present, the comprehensive evaluation mathematical models commonly used in various fields of evaluation have their own characteristics and the application effect is good, but there are also some shortcomings [5]. As can be seen from Figure 1, when the building height is lower than 0, the space utilization will drop sharply. According to the nonlinear characteristics of public building design scheme evaluation and the gradual transitivity of the index system, a three-layer BP neural network is designed. The network includes an input layer, a hidden layer, and an output layer. The input layer has 21 nodes, and the corresponding input vector is set as *X* = (*x*_1_, *x*_2_,…, *x*_21_)^*T*^, which corresponds to 21 evaluation indexes of the evaluation index system of public building design scheme, such as land use environment. The hidden layer has 3 nodes. The output layer has one node, and the corresponding output variable is set to *Y*, which corresponds to the comprehensive evaluation value of public building design scheme [6–9].

Because the research is the co-optimization problem of test time and test power consumption, the genetic algorithm is a global optimization algorithm. SPEA-II algorithm is an excellent multiobjective evolutionary algorithm to study this problem. The essential attribute of residential public space is to meet the needs of residents for travel, and communication. Therefore, strengthening the public space design of residential buildings can not only realize the unified planning of residential buildings but also help to improve the construction level of convenience service infrastructure. At present, people's demand for quality of life is gradually increasing, especially with the continuous advancement of urbanization. The commercialization of housing has also become the trend of the times, in which the design of housing, architecture, and public space is very necessary. It is necessary to fully combine people's specific needs for the interior space of houses, the exterior design of houses, and the corresponding needs to meet people's living needs. Architectural designers also need to reconceive, analyze, and plan the whole design under the guidance of national standards, specifications, and relevant policies, especially for the parts related to room functions and practical uses. Make full use of the geographical environment to rationally organize and collocate the space, and consider the relationship between buildings and people, buildings and environment, and people. Only in this way can we design people-oriented residential houses and create a more comfortable living environment for the majority of households [10]. With the increasing attention paid to public space design, the public space in residential quarters is gradually developing towards refinement and localization. However, in the early design exploration process, there were some problems, such as the uncoordinated scale of residential buildings and residential public space. Because the building area and public space area could not be considered at the same time, the design level only stayed at the minimum standard meeting the requirements of relevant codes. Because of the late start of Chinese urbanization, the lack of unified planning of public space design by government agencies, and the fact that some designers' design ideas have not kept pace with the times, there is an obvious gap between the design effect and the actual demand [11, 12]. In the structure diagram, there can be two input spaces to obtain a result after operation and there is a cyclic joint relationship between the two input and output units. Different from the method in this paper, this paper finds the optimal forecasting scheme based on the neural network combined with the design of the building site [13–15]. This paper builds an accurate and efficient platform for building performance prediction and optimization to help designers make decisions by using a machine learning method.

## 2. The Principle of BP Neural Network and SPEA-II Multiobjective Algorithm

Artificial neural network is a branch of artificial intelligence, which has been used in the fields of model identification and dynamic control. The SPEA-II method is also widely applied to various fields including architectural space design [16, 17]. In addition, in the aspects of information pretest and linear regression, it can also be very effective to use artificial clothes through the network. In the artificial neural network model and algorithm towel, error and backward propagation calculation method is a relatively mature calculation method. The schematic diagram of BP neural network is shown in Figure 2.

The network calculation method is widely used in the fields of pattern recognition, classification, function approximation, and data compression. However, there are still some problems to be solved in the calculation method, which are slower than the collection speed of learning the calculation method through the network, for example, when the calculation is in progress, it is trapped in the local minimum of the prediction office [18, 19]. In view of the shortcomings of the network calculation method of the acupoints, some people have put forward the method of changing and changing the error if the network structure rate of the function and the dynamic adjustment of the parameters to determine the initial value [20]. Theoretically, it has been proved that a network with deviation and at least one type of hidden layer plus a linear output layer can approach any rational number. Increasing the number of layers can further reduce errors and improve precision, but at the same time, it will also make the network complex hybrid, thus increasing the training time of network weights. As can be seen from Figure 3, there is a strong connection between the trained predicted value and the true value. By increasing the number of neurons, the effect of reducing errors and improving precision can be achieved, and the effect of using the number of the cost-making divinatory elements is easier to observe and adjust than increasing the number of layers. The number of neurons in the concealed layer can be given priority if the conditions are allowed [21].

The weight change of neural network in each cycle training is determined by the learning rate. The neural network system will become unstable when the learning rate is high. However, if a small learning rate is adopted, the training time will be prolonged and the convergence rate will be slowed down. If a small learning rate is not adopted, it can ensure that the error of the meridian network is lower than the low valley of the error surface and eventually tends to the minimum error cover value. Under normal cases, the stability of the network system can be ensured by selecting a small learning rate. The learning rate can be chosen from reference [22]. The data collection and standardization of housing construction project is the key point of project parameters, individuals, and personnel. According to the special features of the construction process of the housing project, the information collection standard is divided into two main parts, namely, the basic characteristic information of housing construction and the information of housing construction price. The collection of residential building information mainly includes the name of residential building project, the location of the project, the project category, the information of participants, the time of building, the basis of price calculation, the characteristics of residential building, the characteristics of structure, and decoration. The price information collection includes the price information of construction projects, the cost information of decoration and repair projects, and the cost information of installation projects [23]. In interactive design, from the perspective of reducing information cognitive friction, designers need to take into account the actual operation routes of different user groups in different situations, which are reflected in the logo-oriented system. The information flow line must be made clear, and the target users can be divided into two categories: internal staff and external visitors. Comparatively speaking, the internal staff have a weak demand for the sign-oriented system and the external visitors have a stronger demand for finding the way because they are unfamiliar with the internal environment of the building [24]. Adaptive reuse of interior space is a very effective strategy for sustainable development. However, in practical cases of modern renovation, all design principles and concepts are always based on commercial interests. We can see that “modern ancient town commercial complexes” are springing up like mushrooms after rain, and ancient towns all over the country miraculously achieve uniformity in form and content. This kind of transformation of historical buildings pretends to be twisted under the guise of historical culture and characteristics of the times. Interior design is a combination of the so-called essential elements of different periods, which is neither fish nor fowl nor recognition. Some deliberately exaggerate the historical features, and some swords go astray to seek novelty, completely violating the history and culture of buildings and blocks. This short-sighted behavior should be restrained and criticized.

The SPEA-II algorithm adopts the idea of Pareto, selects the basic idea of the “K-nearest neighbor” algorithm to ensure that the population diversity can be maintained at a high level, and uses the elite retention strategy, and an external dataset is created to temporarily store outstanding individuals. The specific principle and operation process for the SPEA-II algorithm can be found in [25]. The SPEA-II algorithm is a representative elite algorithm in multiobjective optimization algorithms, which have become the performance comparison standards of other multiobjective optimization evolutionary algorithms. The general operation steps of this algorithm are as follows:

1. Initialize population *x*
2. Select the elite solution from *x* to the external set *y*
3. Create a pairing library from either or both *x* and *y*
4. Next generation *x* is created by evolutionary operators based on pairing library reproduction
5. If the external conditions are not met, then go to Step (2)

## 3. Standard Floor Design in Residential Design

### 3.1. Stair Hall Design

The standard floor design in residential design mainly includes public spaces such as staircase halls, corridors, elevator vertical transportation, and so on between floors connected with each household. These areas are the only places for residents, and they are also the most frequently used architectural spaces for residents to communicate with each other. Therefore, designers must pay attention to the design of standard floors [26]:

(1) $$\begin{array}{c} y_{\min}=F\left(x\right)=\left(f_{1}\left(x\right)f_{2}\left(x\right)f_{3}\left(x\right)\ldots f_{m}\left(x\right)\right), \end{array}$$

where *x* is the decision space of *n* dimensions and *y* is the objective vector of *m* dimensions.

Because of the differences in residential construction age and design, stair hall design can be divided into two ways: traditional low-floor walking stairs and high-rise elevator design. Stairs and elevators constitute the vertical transportation system in residential buildings. First, designers should design public space separately from the characteristics of two different traffic forms. Second, designers should have a full understanding of these two vertical transportation modes because they are very important for building a harmonious neighborhood relationship [27, 28].  Figure 4 shows the two sets of parallel sequences are not significantly different in value. Therefore, the calculation results are feasible. It shows that if the design is improper or the design parameter standards are not in line with the reality, users will often stop for a long time, which will have a negative impact on building the neighborhood relationship. Third, with the increase of high-rise buildings, the elevator hall has become an important place for residents to communicate with each other. Designers should strengthen the design of safety facilities in stairwells and fire escape routes to ensure the safety of residents' lives and property.

### 3.2. Corridor and Roof Design

Figure 5 shows the neural network training diagram. When designing the corridor, the designer should start from meeting the needs of multiple households and reflect the utilization value of the corridor in the design process. Second, we should change the traditional design pattern. For example, there are a large number of households in corridor-style houses, lack of recognition, and it is easy to go wrong without the help of doorplate signs [29, 30]. The MRE calculation formula is as follows:

(2) $$\begin{array}{c} MRE=\frac{1}{N}\sum_{i=1}^{n}\frac{\left|Y_{i}-P_{i}\right|}{Y_{i}}. \end{array}$$

This function is used to characterize the error level between the true value of the whole sample and the prediction.

First, the roof layer design should be taken seriously as an important part of the public space of residential buildings, fully embodying the function of roof heat insulation and rain protection and reducing the probability of rainwater leakage on the roof. Second, the design should first consider the practical function of the roof, ensure that vertical transportation systems such as elevators can reach the roof, meet the basic needs of residents, and reserve working space for repair and maintenance. It can be seen from the structure diagram in Figure 6 that the algorithm has a strong mapping relationship. Third, it shows that, in the process of roof traffic design, it is necessary to scientifically select materials such as heat insulation, cold protection, and leakage prevention and the materials used should meet the requirements of energy conservation and environmental protection. Fourth, the shape and color of roof design in residential building design should be unified and coordinated with the same residential area and surrounding residential areas, reflecting the beauty of harmony.

(3) $$\begin{array}{c} R^{2}=\frac{\sum_{i=1}^{n}\left(P_{i}-\overset{¯}{P}\right)\left(Y_{i}-\overset{¯}{Y}\right)}{\sqrt{\sum_{i=1}^{n}{\left(P_{i}-\overset{¯}{P}\right)}^{2}}\sqrt{\sum_{i=1}^{n}{\left(Y_{i}-\overset{¯}{Y}\right)}^{2}}}. \end{array}$$

In the above formula, *Y*_i_ is the true value of the *i*th sample and *I* is the predicted value of the *i*th sample.

In the design of the central green space of residential buildings, the following requirements should be adopted: first, green the construction green space in the central area with enclosed layout; second, the design of central green space should fully consider the actual needs of residents, take flowers, shrubs, and other low plants as the main body according to the pH value of land and soil, and appropriately decorate the garden with landscape sketches to improve the aesthetics of central green space; third, in order to ensure the integrity of the central green space design of residential buildings, the central green space should be combined with daily departure routes such as roads and landscape trails in residential areas.

(4) $$\begin{array}{c} N_{j+1}=\left(A\times N_{j}+B\right)\mathrm{mod}\left(M\right), \end{array}$$

where *A* is the multiplier, *B* is the increment, *M* is the modulus, and mod is the remainder algorithm.

The divergence problem is the weight nonconvergence problem in the process of adaptive filtering, which is generally caused by the misalignment of the reference signal and the near-field data. In the process of error elimination, the residual error should be monitored. If the residual value exceeds the data of near-field monitoring, divergence phenomenon will occur. At this time, the residual signal should be modified to achieve convergence of calculation.

### 3.3. Architectural Space Design under the Integrated Space Model

In recent years, the space design under the integrated space model has been widely used in commercial and exhibition space, and it is an expression of immersive space. The integrated space design pays attention to the interaction and integration between people and the environment, that is, it is used to integrating people's emotions into the architectural environment, which is more dependent on the creation of landscape environment space. Usually, people's walking path and the expression of space are integrated with each other by using the introduced design method, so as to introduce the feeling of walking space experience into the external space environment:

(5) $$\begin{array}{c} I_{cz}=\frac{\sum_{i=1}^{n}B_{oi}C_{oij}}{\sum_{i=1}^{n}B_{i}C_{ij}}, \end{array}$$

where *I*_cz_ is the correction coefficient.

The integrated space is often used in the design of exhibition buildings, and the external landscape space and atmosphere are often used to create a sense of enclosure between places, which closely combines the walking path of people with the landscape. One side of the corridor is enclosed by a stone wall, the other side is completely empty, and the borderless space design is carried out. When people are in the corridor, they can feel that the overall space atmosphere is almost integrated with people's walking path. At the same time, in the design, the screen is used to properly block, define the landscape and gray space, and highlight the continuity of the integrated space.

(6) $$\begin{array}{c} J=\overset{P}{\underset{p=1}{\sum }}\left(0.5\overset{n}{\underset{j=1}{\sum }}{\left(t_{pj}-o_{pj}\right)}^{2}\right), \end{array}$$

where *j* represents the total error function of BP network training.

The integrated space design focuses on people's perception and analysis of the surrounding environment during walking and makes the surrounding environment landscape play a role in guiding people's behavior or generating interaction with people. Around buildings and waterscapes, a large area of landscape water surface is used to create and design the overall space atmosphere, a narrow path is designed for passage on the water surface, and the periphery of the path is designed without boundary, so that people's walking and the overall space atmosphere are integrated with each other, so as to strengthen the interaction between people and waterscapes and people and buildings and break the sense of emptiness and fierceness of the overall space. At the same time, trees and other markers are used in the middle of the path to highlight the landmark in the space, so as to realize the guiding role of landscape space to the external environment.

(7) $$\begin{array}{c} △=\sqrt{\frac{1}{m-1}\sum_{i=1}^{m}{\left(\overset{¯}{S}-S_{i}\right)}^{2}}, \end{array}$$

where *S*_i_ is the minimum distance between the *i*th noninferior solution and other noninferior solutions in multidimensional space.

The integrated space model is also often used in the entrance and exhibition of commercial buildings. It pays more attention to the transformation of space scale, and it is customary to integrate the traveling experience into the commercial building space by the way of piecemeal design.  Figure 7 shows that the efficiency of the third fitting curve is higher than the other three, so it can be selected as our impact factor. At the entrance of the building, oblique spatial organization is adopted to introduce large-scale space into small-scale space, and at the same time, a large-area glass surface is adopted around the building to form an immersive entrance space experience. In the ceiling of the building, vertical slices are used for guidance and the sense of movement in the space is integrated into the entrance space of the building, which is naturally combined into a part of the integrated space model. The adopted algorithm changes the values of relevant variables one by one, so as to explain the law of how the key indicators are affected by these factors. Therefore, there is no sensitivity analysis in the process of realizing the algorithm function.

## 4. Selection of Characteristic Parameters of Architectural Design

The SPEA-II algorithm has been improved in the fitness assignment method, and a new environment selection strategy is adopted. The new environment selection strategy is based on the characteristics of proximity rules, so that the solution set obtained by the SPEA-II algorithm is superior to other algorithms. Distribution uniformity, especially in solving high-dimensional optimization problems, is an important factor of calculation. Nine important parameters in spatial design are used as the inputs of neural network, which are the spatial category, spatial degree, site category, spatial grouping, aspect ratio, aspect ratio, total mass, bottom stiffness, and bottom area. The aspect ratio, total mass, bottom stiffness, and bottom area are different in numerical ranges and units, so the data must be normalized by [−1, 1] before input, so that the input components can be trained in the form of dimensionless network, and at the same time, the phenomenon of neuron output saturation caused by excessive absolute value of net input can be avoided. Normalization processing formula is

(8) $$\begin{array}{c} \overset{¯}{x_{i}}=\frac{2\left(x_{i}-x_{\min}\right)}{x_{\max}-x_{\min}}-1, \end{array}$$

where *x*_i_ represents input data and *x*_max_ represents the maximum value in the data.

MATLAB 6.5 neural network toolbox is used to establish BP neural networks isolat-network1 and isolat-network2, which are used to test the maximum displacement of the support under the action of the maximum story shear ratio of the structure. Both neural networks, isolat-network1 and isolat-network2, use momentum gradient descent method to adjust network weights and thresholds. In this neural network, the number of neurons in the input layer is 7, the number of neurons in the hidden layer is 10, and the number of neurons in the output layer is 4. The neurons in the input layer adopt linear transmission, and the neurons in the hidden layer and the neurons in the output layer all adopt tangent sigmoid function.

(9) $$\begin{array}{c} D=\sqrt{\overset{M}{\underset{m=1}{\sum }}{\left(\max f_{m}^{i}-\min f_{m}^{i}\right)}^{2}}, \end{array}$$

where *m* is the target dimension and *D* is a nondominant set.

The training of neural network divides 40 design samples into two groups: 25 samples in group A are neural network training samples and 15 samples in group B are neural network test samples. The neural network isolat-network1 is used to test the maximum utilization rate of space. The network inputs are the spatial category, spatial degree, site category, spatial grouping, aspect ratio, length-width ratio, total mass, and bottom stiffness of the building. The backpropagation algorithm based on Levenberg–Marquardt optimization theory is used to train the network. The training error target value is 1 × 10^−5^, isolat-network1 meets the error requirement when the training reaches the 12th step, and the training ends. The neural network isolat-network2 is used to test the maximum displacement of the structure on the support. It can be seen from Figure 8 that the fault tolerance rate is negatively correlated with the increase of the unique value. The network inputs are the spatial category, spatial degree, site category, spatial grouping, aspect ratio, aspect ratio, bottom stiffness, and quality per unit area of the bottom. The backpropagation algorithm based on Levenberg–Marquardt optimization theory is used to train the network. The training error target value is 1 × 10^−5^, isolat-network2 meets the error requirement when the training reaches the 23rd step, and the training ends.

## 5. Landscape and Regional Spatial Layout Design

The SPEA-II algorithm adopts a new fitness assignment method that combines the fine-grained original fitness assignment method and the density estimation method. For each individual, the assignments influence their dominance. In the architectural landscape, the spatial sequence of multiviewpoint and multispace changing scenes is reflected and a picturesque garden sketch is constructed by combining green plants, artificial water bodies, corridors, and bridges. China's landscape design has a long history, and its aesthetic art is closely related to splendid Chinese literature, art painting, and poetry. The application of traditional artistic creation methods and concepts in the process of architectural landscape and regional spatial layout design, such as the scattered perspective method in landscape paintings and the artistic concept of “stone divided into three sides” in Chinese painting art, will effectively increase the aesthetic interest of landscape design.

(10) $$\begin{array}{c} \varphi \left(x\right)=\frac{1}{x+\sqrt{x^{2}+\varepsilon^{2}}}, \end{array}$$

where *ε* is a constant that is not very small.

The emblem-style architectural style with black and white walls, the patchwork of green plants and pots, and the twists and turns of antique stone roads form a leisurely artistic conception of space. In the design process, it is particularly important to make the plaques and lights in the building decorate according to the overall landscape atmosphere and to build a complete space artistic conception.  Figure 9 shows that the component value exhibits periodic changes and has gradually become denser in recent years. For different architectural community styles, the foothold of landscape planning and design is often different. The details of the landscape around the building need special attention. Only by ensuring the unity of the overall shape and aesthetics can we achieve the integration between the building and the landscape, enhance the rhythm of the overall space, and ensure the integrity. If the buildings adopt the industrial paradigm of cold-tuned light source, then this artistic conception will be greatly reduced.

The layout design of landscape and regional space follows western art design ideas, and under the concept of minimalism, a small number of design elements are selected to develop landscape space. Take a single landscape with a sense of design as the visual center, so as to lay out green plants and waterscapes, make full use of natural energy, and build a leisure space with ecological characteristics. Western art ideas and creative techniques are also often applied to architectural landscape design, which mainly pursues the design concept of people-oriented and nature-oriented and creates a simple and comfortable space atmosphere with very pure design.

(11) $$\begin{array}{c} E_{p}=\sum_{s_{i}}e^{s\left[{\left(c_{i}-c_{s}\right)}^{2}-R\right]}. \end{array}$$

In the formula, *c*_s_ is the center position of *s*_i_ after uniform shrinkage and expansion.

The chic seat is very modern, with special materials, uniform color and floor decoration, and simple and fresh style. Rest area is a very important link in architectural landscape and spatial layout design. In the design process of this functional area, special architectural sketches with special seats, pavilions, corridors, flower stands, sculptures, signboards, etc. can be generally used to enhance the artistic charm of regional space. In this kind of architectural sketch design process, we should balance the economy and aesthetics not only to ensure the harmony and unity between these architectural sketches and architectural landscape but also to pay attention to the economic cost of relevant materials with modeling characteristics and aesthetic characteristics of the times. New environmental protection materials can be appropriately introduced to create new visual effects to build a more eye-catching landscape area.

## 6. Data-Driven Layout Design of Indoor Space

Layout plan design is an important part of residential building because layout plan is the design blue plan of residential building, which reflects the type, square position, size, adjacent relationship, and wall distribution of rooms in the room layout. General layout plan design usually requires the indoor designers to go through repeated tests and groping, and a great deal of professional knowledge and design experience are needed, so layout plan design is a time-consuming process. The purpose of our research is to make this design process self-moving and to design a reasonable indoor space layout for residential buildings automatically and efficiently.

(12) $$\begin{array}{c} E\text{ size}={\sum \left(w_{i}-w^{\prime }\right)}^{2}+{\left(d_{i}-d^{\prime }\right)}^{2}, \end{array}$$

where *w* and *d* are the width and height of the target room, respectively.

BP neural network technology can automatically and effectively generate the indoor layout plan of residential buildings with given boundary.  Figure 10 shows that we have constructed a large-scale dataset Rplan, which includes more than 80,000 indoor layout plans from real houses. Each layout plan in the dataset is represented as a vector figure with detailed label. In design practice, an important observation is that designers mainly adopt two-step strategy to design the layout of rooms: they first determine the relationship and position of rooms and then calculate the size of rooms and the position of walls. Inspired by the design process of indoor space layout by designers, we put forward a two-stage generation algorithm of indoor space layout, that is, first locate the location of rooms and then determine the location of walls. In order to pretest the layout of rooms, we learned from the new learning methods and combined with the priority positioning strategy of the guest room to improve the rationality of the layout design. In this step of positioning the wall, based on the predicted room position, we first use a network of coders and decoders to predict the position of the wall and then use some postprocessing operations to convert the layout plan into the final vector grid.

At present, our method only focuses on the layout plan of single-storey residential building design. For multistorey residential buildings, it is necessary to connect two consecutive floors through stairs. Generally speaking, the stairs are expressed as a special type of room, but the direct connection should use our method. First, we created the layout plan of the first floor including stairs, and then we created the layout plan of the second floor according to the layout plan of the first floor. The stairs built in the first floor should be used as the design constraint for building the second floor layout. However, in the real world, stairs have a special shape and location. For our deep network, it is difficult to control the generation of stairs. In addition, even if no guest room is located first, our second-order section method can also be extended to other types of layout design, such as writing word floor, shopping center, and supermarket, but before that, we must have relevant data. We believe that this model has certain applicability in current architectural design research. However, a limitation of this approach is the lack of much validation for future more complex building structures.

## 7. Conclusion

In view of the complexity of the comprehensive evaluation of public building design schemes and the nonlinear relationship among influencing factors, this paper analyzes two main problems existing in the current comprehensive evaluation methods. This paper designs a general evaluation model for evaluating various public building design schemes and constructs an evaluation model based on the improved BP neural network algorithm. Furthermore, the evaluation model and algorithm based on self-organizing competitive neural network are proposed and applied to an example. After solving and verifying, it is shown that the theories and algorithms of these two neural network evaluation models are reasonable and effective in algorithm and are suitable for comprehensive evaluation of public building design schemes. It can basically solve the main problems existing in the previous comprehensive evaluation methods and reduce the subjectivity existing in each stage of the comprehensive evaluation process. In summary, this paper builds an accurate and efficient platform for building performance prediction and optimization to help designers make decisions combined with a BP neural network and the SPEA-II multiobjective optimization algorithm. Compared with other research group works, the optimization results of the case are quantitatively and qualitatively analyzed and presented in visual form based on the BP neural network prediction model. In the design of public space in residential buildings, we should firmly grasp the main purpose of providing residents with good public communication, public activities, and leisure and entertainment places, embody the principle of people-oriented, green home, and overall consideration, and create high-quality public space design products in residential buildings according to the specification requirements of standard floor design, so as to create good conditions for improving residents' quality of life. Therefore, the biggest contribution of this study is that it proposes a method and idea of green building energy-saving design. This work will help popularize machine learning in architectural design around the world.

## Figures and Tables

**Figure 1:** Building-level spatial data.

**Figure 2:** Principle of neural network calculation.

**Figure 3:** Comparison between real value and predicted value.

**Figure 4:** Comparison of two groups of parallel data. Parallel coordinates' plot of (a) the first set of random data and (b) the second set of random data.

**Figure 5:** Neural network training diagram.

**Figure 6:** Neural network structure diagram.

**Figure 7:** BP neural network training effect.

**Figure 8:** Relative error diagram.

**Figure 9:** Influence of temperature, displacement, and human factors with time.

**Figure 10:** BP network neural prediction trend chart.

## Data Availability

The data used to support the findings of this study are available from the corresponding author upon request.
